# Quantitative Evaluation of Plant and Modern Urban Landscape Spatial Scale Based on Multiscale Convolutional Neural Network

**DOI:** 10.1155/2021/7742700

**Published:** 2021-07-22

**Authors:** Yang Wang, Moyang Li

**Affiliations:** ^1^School of Design & Art, Xijing University, Xi'an, Shaanxi 710123, China; ^2^No. 705 Research Institute, CSIC, Xi'an, Shaanxi 710077, China

## Abstract

Modern urban landscape is a simple ecosystem, which is of great significance to the sustainable development of the city. This study proposes a landscape information extraction model based on deep convolutional neural network, studies the multiscale landscape convolutional neural network classification method, constructs a landscape information extraction model based on multiscale CNN, and finally analyzes the quantitative effect of deep convolutional neural network. The results show that the overall kappa coefficient is 0.91 and the classification accuracy is 93% by calculating the confusion matrix, production accuracy, and user accuracy. The method proposed in this study can identify more than 90% of water targets, the user accuracy and production accuracy are 99.78% and 91.94%, respectively, and the overall accuracy is 93.33%. The method proposed in this study is obviously better than other methods, and the kappa coefficient and overall accuracy are the best. This study provides a certain reference value for the quantitative evaluation of modern urban landscape spatial scale.

## 1. Introduction

With the rapid development of urbanization in China, the landscape area is shrinking, which has a serious impact on the sustainable development of ecology in China [1]. It is of great significance to grasp the spatial scale of urban landscape in time for the development and protection of landscape [2]. At present, remote sensing image technology has been widely used in landscape resources monitoring due to its advantages of wide coverage, fast acquisition speed, and large amount of information data [3]. The key of plant garden monitoring technology is the extraction of remote sensing images. However, because of the large amount of image data information, traditional technology cannot meet the current requirements of image information extraction, resulting in low precision after extraction [4]. How to extract the information from the remote sensing image of plant garden has become a hot spot in this field. At present, there are many new methods about image information extraction, in which deep learning is the most widely used method in information extraction technology [5]. The learning method is originated from machine learning, including multi hidden layer network mechanism, has strong feature learning ability, and has a great advantage in image classification. Therefore, based on the application of deep learning method, this study combines spectral characteristics and spatial information to extract plant garden information, aiming to provide a basis for modern urban landscape planning [6].

With the development of deep learning, convolutional neural network has become the most popular one in many models in recent years. Thangaraj et al. [7] proposed a deep convolutional neural network model based on transfer learning, which is used to identify tomato leaf diseases and to detect disease by real-time images and stored tomato plant images. The experimental results show that the model is effective in automatic classification of tomato leaf diseases. Ghorbanzadeh et al. [8] used the deep learning convolutional neural network (CNN) to study the influence of optical data from PlanetScope sensor and terrain factors from ALOS sensor on EQIL mapping. The results show that the training data set of spectral information and the terrain factors of slope can help to distinguish the landslide body from wasteland and other similar features, thus improving the mapping accuracy. Paul et al. [9] proposed a hybrid evolutionary network structure search method, proposed the target convolution class of neural network, and proposed a high efficiency representation of the network of fine string representation method and sparse block evolution into dense network necessary hierarchical characteristics concept, and in the medical field to verify various benchmark data sets. Srinivasan and Senthil Kumaran [10] designed a deep convolutional neural network model for superresolution weld image to determine the trace of intermetallic compounds and detect the damage on the weld surface. Zhou et al. [11] put forward a small MBConv block to improve the network model, which makes the network have less training parameters, effectively reduces the problem of over fitting, and improves the classification performance compared with the original model. The results show that the average accuracy of the model to multi classification is 95.78%, which is 2.19% higher than the original model. Sulthana et al. [12] introduced the recommendation system with product visual characteristics, and through a deep architecture and a series of convolution operations, the edges and bubbles in the image overlap. The experimental results show that the image quality of the method is better than that of the weld image generated by the double cubic interpolation method. Wang et al. [13] proposed an integrated convolutional neural network (CNN) to identify and classify four kinds of fuzzy images: defocusing, Gaussian, smoke, and motion. In each stage, deep CNN is used to extract image features, which overcomes the disadvantages of poor scalability and complexity of calculation. The experimental results show that the model has good performance in mutation and gradient detection. Han et al. [14] studied and compared the target recognition effects of two convolutional neural network models, which are fast *r*-CNN and SSD, and evaluated by using average accuracy (map). The results show that there are three types of *r*-CNN with fast speed, with an accuracy of over 80%, SSDs of 7 types and accuracy of over 80%, all of which have achieved good results. Wang et al. [15] proposed a method based on deep convolutional neural network. Using VGGA, VGG16, Perception V3, ResNet50, and CPAFnet, the deep neural network model designed in this paper, the pest image was identified by triple verification method on the CPAF data set. The results show that the results of the model optimization and the CPAFnet depth model for CPAF data set have a good practical significance for intelligent identification of agricultural and forest pests. Linda et al. [16] proposed a color-mapped contour gait image (CCGI). The first contour in each gait image sequence is extracted by the CORF contour tracking algorithm. The algorithm uses the difference of Gaussian (DoG) and the threshold of lag to extract the contour image. Finally, the performance analysis of CVGR is evaluated by using the deep convolutional neural network (CNN) framework. The results show that the accuracy of the method is 94.65%. It is found that when dimension problem is processed, the extracted feature can represent the image quality well. After comparing the influence of different linear and nonlinear reduction techniques on the characteristics of convolutional neural network, a completely image-based recommendation model is established. Wang et al. [17] proposed a multistage camera boundary detection framework based on deep CNN. The process consists of three phases, including candidate boundary detection, mutation detection, and gradient detection. The numerical experiments show that the method has better performance than the previous AlexNet and Google network and other advanced methods. The impact of deep learning is not limited to the field of computer vision and artificial intelligence, such as face recognition, speech recognition, and so on. It plays an important role in the Internet-based service industry in the era of big data. For example, the data intelligence in the field of search engine is an important field in which the major giants are competing to invest in research.

In conclusion, a large number of scholars have studied and applied the deep convolutional neural network in various fields. In view of this, this paper proposes a model of plant and modern urban landscape spatial scale evaluation based on deep convolutional neural network, which can provide some reference and reference for urban landscape planning.

## 2. Extraction of Landscape Information Based on Deep Convolutional Neural Network

### 2.1. Multiscale Convolutional Neural Network Classification Method for Landscape Architecture

Deep learning is a hot topic in the field of machine learning in recent years, and its model structure has more depth than shallow learning. The common models are divided into three structures: hybrid, discriminative, and generative depth, mainly restricted Boltzmann machine (RBM), sparse coding (SC), depth automatic encoder (DAE), depth belief network (DBN), and convolutional neural network (CNN) [18, 19]. Among them, CNN model is widely used in deep learning. Its main advantage is that it has shared weights, which makes the network structure have fewer parameters. Secondly, CNN contains pooling layer, which can ensure that the translation and rotation of the model are not deformed when training learning data. Therefore, this study will apply CNN to classify multiscale landscape.

The traditional CNN method belongs to a hierarchical neural network structure for feature extraction. In this study, the receptive field of image data with constant size is set in advance, and then it is imported into CNN to extract information features, as shown in Figure 1.

Generally, the feature map of layer *l* convolution layer is generated by *l* − 1 layer through a trainable filter *k* and importing the trained data into the activation function SIGMOD function *g*(*x*)=(1+*e*^−*x*^)^−1^ to generate the output data of layer *l* convolution layer. The calculation of layer *l* convolution layer *C*^*l*^ is shown in the following formula:

(1) $$\begin{array}{c} C^{l}=g{\left(k^{l}h^{l-1}+b^{l}\right)}^{-1}. \end{array}$$

In equation (1), *b*^*l*^ is the offset of the *l* layer convolution layer feature map, *h*^0^ is the initial input data, and *h*^*l*−1^ is the *l* − 1 layer hidden layer. In the convolution layer training process, each convolution kernel *k* will cover all the image data to form a feature map, and the convolution layer is the optimal filter for autonomous learning and selection [20]. The subsampling layer samples and extracts through the feature layer to reduce the difficulty of training and learning, greatly reducing the feature layer and making the training process more stable [21]. The definition of subsampling layer is shown in the following equation:

(2) $$\begin{array}{c} S^{l}=g\left(\text{down}\left(h^{l-1}\right)+b^{l}\right). \end{array}$$

In equation (2), down() is a subsampling function, and *n* × *n* region is usually used to process the input data, so that the input feature map is *n* times smaller than before. The output data are given the bias parameter *b*^*l*^, so that the features with correlation are extracted layer by layer.

CNN usually extracts spatial related elements from a fixed size range, which limits the observation scale, resulting in low image classification accuracy [22]. In order to improve the accuracy, it is necessary to extract multiscale spatial elements. Firstly, the pyramid algorithm is applied to obtain images of different observation scales, and all data are input into the network structure for information feature extraction [23]. In the initial *M* band {*I*_*m*_}_*m*=1_^*M*^, the pyramid image set {*P*_*s*_}_*s*=1_^*S*^ with parameter *S* is constructed, in which the first scale {*P*_*s*_}_*s*=1_^*S*^ is the same as band *I*_*m*_, and *P*_*s*_^*m*^ can be obtained on the basis of *P*_*s*=1_^*m*^. If there is a multiscale training sample {*X*^*n*^}_*n*=1_^*N*^ with *C* categories, the square sample set generated by receptive field is represented by *X*^*n*^, and the reference pixel set is represented by label. The structure process of multiscale CNN learning and training is shown in Figure 2.

The *L*-layer network structure in Figure 2 is the bias vector *b* and the learning filter *k* of the square error cost function. The forward propagation cost function is shown in the following equation:

(3) $$\begin{array}{c} \min\ell \left(k,b\right)=\frac{1}{2}\overset{N}{\underset{n=1}{\sum }}\left(t^{n}-y^{n}\left(k,b\right)\right)=\frac{1}{2}\overset{N}{\underset{n=1}{\sum }}{\left\|t^{n}-y^{n}\left(k,b\right)\right\|}_{2}^{2}. \end{array}$$

In equation (3), *y*^*n*^(*k*, *b*) is the prediction label of multiscale CNN for sample *X*^*n*^ and *t*^*n*^ is the training sample *X*^*n*^ of *n*. *h*^*l*^ is used to represent the hidden layer of layer *l*, and *l* ∈ {1,2,3,…, *L*}, *h*^0^ are the input raw data. The output layer is obtained as shown in the following equation:

(4) $$\begin{array}{c} y\left(k,b\right)=g\left(a^{L}\right),\;a^{L}=k^{L}h^{L-1}+b^{L}. \end{array}$$

The label values of reference and output are compared, and the bias vector and filter parameters are optimized by random gradient descent method. The multiscale CNN spatial feature elements are obtained as shown in the following equation:

(5) $$\begin{array}{c} F=f\left(k,b|X\right)=g\left(kX+b\right). \end{array}$$

Multiscale CNN can obtain multiscale spatial feature elements from samples and can optimize bias vector and filter parameters by using back-propagation algorithm. Its nonlinear features play a greater role in target recognition and classification [24]. The context scenes of different sizes are imported into the multiscale feature learning, and several CNN models are run. Finally, all the outputs are merged into the full connection layer. The process of pixel classification in remote sensing image using a single CNN is shown in Figure 3.

Remote sensing image (*m*) in CNN input layer × *m*: there are *C* bands, and the classified pixels are located in the center. The *L* subsampling layer in CNN is connected with the standard convolution layer and connected to the full connection layer. The first CNN layer includes subsampling layer and convolution layer. After pooling, feature elements are obtained. Then, nonlinear function activation and local standardization are performed. Then, the output subsampling layer data of the last layer is imported into the fully connected layer. Finally, the output data of the fully connected layer is imported into the softmax classifier to obtain the final classification result [25].

Figure 4 shows the structure of multiscale CNN model. In Figure 4, there are *n* CNN parallel operations and *l* convolution and pooling processes, and the context scene scale is 1 m∼nm. The output of each CNN is connected to the full connection layer, and the output of the full connection layer is the input of the classifier to ensure that the parameter training of each CNN is consistent with the pixel-by-pixel learning training of a single CNN.

### 2.2. Construction of Landscape Information Extraction Model Based on Multiscale CNN

Firstly, the normalized difference water body index (NDWI) of landscape is calculated, which is mainly used to calculate the specific bands in remote sensing data, suppress vegetation and other information through the ratio of near-infrared band and green light, and enhance the display of information features in the image. The formula is shown in the following equation:

(6) $$\begin{array}{c} \text{NDWI}=\left\{\begin{array}{cc} \frac{G-\text{NIR}}{G+\text{NIR}}, & G\geq \text{NIR},\\ 0, & G<\text{NIR}. \end{array}\right. \end{array}$$

In equation (6), NIR and *G* are near infrared band and green band images, respectively.

Figures 5(a) and 5(b) are the original images of true color band combination of remote sensing image and the gray image after NDWI index calculation, and the water information in the image after calculation is more obvious.

Then, the linear tassel cap transform (*K*-*T* transform) is used to transform the spectral features into the new feature space, and the four band orthogonal transform is used to transform the image, and the plant spectrum will be hat-like distribution. *K*-*T* transform can reduce the influence of spectral characteristics between ground objects in spectral remote sensing image. The transformed band gray value *u* is shown in the following equation:

(7) $$\begin{array}{c} u=R^{T}x+r. \end{array}$$

In equation (7), *r* is the offset, *x* is the gray value of each band, and *R* is the coefficient of *K*-*T* transform. The multispectral remote sensing image after *K*-*T* transform includes three components: brightness, greenness, and humidity. The humidity component (*KT*3) has more reference value, which can effectively reflect the distribution of surface moisture content.  Figure 5(c) is the humidity distribution map obtained by *K*-*T* transformation in Figure 5(a), and the calculated flow area information is obvious. Then, the fractal network evolution method (fnea) is used to segment the image data, and the optimal segmentation parameters are selected to segment the image data.

Then, the data samples of rivers, lakes, cultivated land, constructed wetlands, and construction land are selected to construct the multiscale CNN landscape information extraction model. Remote sensing training image data selection 32 × 32, 64 × 64, 128 × 128, multiscale CNN consists of 9 layers, including input layer, 3 convolution layers, 3 sampling layers, full connection layer, and output layer. The structure of multiscale CNN is shown in Figure 6.

As shown in Figure 7, the figure shows the characteristic map of each training sample, such as river, swamp, constructed wetland, etc. At the same time, taking the river in the feature map as an example, Figure 6 shows the feature subgraphs of the data samples from the input layer to the convolution layer and the sampling layer.

Fnea is used to segment the NDWI gray image, and then the average value $\bar{\text{NDWI}}$ of each spot is calculated. The calculation method of water probability based on NDWI is constructed, as shown in the following formulae:

(8) $$\begin{array}{c} {\bar{\text{NDWI}}}_{j}=\frac{1}{n}\overset{n}{\underset{i=1}{\sum }}{\text{NDWI}}_{i}, \end{array}$$

(9) $$\begin{array}{c} P_{j}^{\text{NDWI}}=\frac{{\bar{\text{NDWI}}}_{j}-{\bar{\text{NDWI}}}_{\min}}{{\bar{\text{NDWI}}}_{\max}-{\bar{\text{NDWI}}}_{\min}}. \end{array}$$

In equations (8) and (9), *n* is the number of pixels in the image spot, *i* and *j* are the *i* − th pixel of the image spot and the *j* − th image spot, ${\bar{\text{NDWI}}}_{\min}$ and ${\bar{\text{NDWI}}}_{\max}$ are the minimum and maximum values of the image spot, respectively, and *P*_*j*_^NDWI^ is the probability that the *j* − th image spot is a water body. Then, the segmented patches are imported into the multiscale CNN recognition model to obtain the recognition probability *P*_*j*_^DCNN^. Multiscale CNN can be expressed as *y*=[*y*_1_, *y*_2_,…, *y*_*m*_], and ndmi can be expressed as *x*=[*x*_1_, *x*_2_,…, *x*_*m*_], where *m* is the number of spots, and the calculation of joint probability *P*_*j*_^water^ of spatial spectrum of water body is shown in the following equation:

(10) $$\begin{array}{c} P_{j}^{\text{water}}=p\left(x_{j}\cap y_{j}\right)=p\left(x_{j}\cap y_{j}\right)p\left(y_{j}\right)=P_{j}^{\text{DCNN}}*P_{j}^{\text{NDWI}}. \end{array}$$

The higher the accuracy of combining multiscale CNN and ndmi to calculate the water target, the greater the *P*_*j*_^water^ value. The weighted average method is used to calculate the joint probability center of spatial spectrum, and the water spots with higher probability are introduced into the joint probability interval of spatial spectrum, and the convergence is continued until the best effect of water target recognition is achieved. Finally, the joint probability weighted center *P*_mean_^water^ of spatial spectrum is calculated, and the method is shown in the following equation:

(11) $$\begin{array}{c} P_{\text{mean}}^{\text{water}}=\frac{1}{m}\overset{m}{\underset{j=1}{\sum }}P_{j}^{\text{water}}*W_{j}. \end{array}$$

In equation (11), *W*_*j*_ is the weight of the *j* spot, and the formula is *W*_*j*_=((*e*^*P*_*j*_^water^^ − 1)/∑_*i*=1_^*m*^[*e*^*P*_*j*_^water^^ − 1]). The calculation of mean square error *P*_std_^water^ of joint probability of space spectrum is shown in the following equation:

(12) $$\begin{array}{c} P_{\text{std}}^{\text{water}}=\sqrt{\frac{1}{m}\overset{m}{\underset{j=1}{\sum }}{\left(P_{j}^{\text{water}}*W_{j}-P_{\text{mean}}^{\text{water}}\right)}^{2}}. \end{array}$$

If |*P*_*j*_^water^*∗W*_*j*_ − *P*_mean_^water^| > 3*∗P*_std_^water^, the pattern spot will be removed, and the error will be recalculated by returning equations (11) and (12) until the calculation result converges. Continue to segment the gray image of humidity component, and calculate the mean value $\bar{\text{KT}3}$ of KT3 to construct the landscape probability map based on KT3, as shown in the following equations:

(13) $$\begin{array}{c} {\bar{\text{KT}3}}_{j}=\frac{1}{n}\overset{n}{\underset{i=1}{\sum }}\text{KT}3_{i}, \end{array}$$

(14) $$\begin{array}{c} P_{j}^{\text{KT}3}=\frac{{\bar{\text{KT}3}}_{j}-{\bar{\text{KT}3}}_{\min}}{{\bar{\text{KT}3}}_{\max}-{\bar{\text{KT}3}}_{\min}}. \end{array}$$

In equations (13) and (14), *P*_*j*_^KT3^ is the probability that the *j* spot of KT3 is a wetland and ${\bar{\text{KT}3}}_{\max}$ and ${\bar{\text{KT}3}}_{\min}$ are the maximum and minimum values of KT3 in the image, respectively. If KT3 is represented by *z*=[*z*_1_, *z*_2_,…, *z*_*m*_] and *m* is the number of patches, then the joint probability *P*_*j*_^wetness^ of wetland spatial spectrum is calculated as shown in the following equation:

(15) $$\begin{array}{c} P_{j}^{\text{wetness}}=p\left(z_{j}\cap y_{j}\right)=p\left(z_{j}\cap y_{j}\right)p\left(y_{j}\right)=P_{j}^{\text{DCNN}}*P_{j}^{\text{KT}3}. \end{array}$$

The space spectrum joint probability weighting center *P*_mean_^wetness^ is shown in the following equation:

(16) $$\begin{array}{c} P_{\text{mean}}^{\text{wetness}}=\frac{1}{m}\overset{m}{\underset{j=1}{\sum }}P_{j}^{\text{KT}3}*W_{j}. \end{array}$$

In equation (16), *W*_*j*_ is the patch weight of the *j* graph, and the formula is *W*_*j*_=((*e*^*P*_*j*_^wetness^^ − 1)/∑_*i*=1_^*m*^[*e*^*P*_*j*_^wetness^^ − 1]). The error *P*_std_^wetness^ of joint probability weighting center of space spectrum is shown in the following equation:

(17) $$\begin{array}{c} P_{\text{std}}^{\text{wetness}}=\sqrt{\frac{1}{m}\overset{m}{\underset{j=1}{\sum }}{\left(P_{j}^{\text{wetness}}*W_{j}-P_{\text{mean}}^{\text{wetness}}\right)}^{2}}. \end{array}$$

If |*P*_*j*_^wetness^*∗W*_*j*_ − *P*_mean_^wetness^| > 3*∗P*_std_^wetness^, the spot is removed and the error is calculated repeatedly until the result converges.

## 3. Quantization Effect Analysis of Deep Convolutional Neural Network

### 3.1. Training Effect of Convolutional Neural Network

In this study, a city garden wetland landscape is selected for research. Firstly, the landscape area is classified into seven categories, including construction land, bare land, constructed wetland, cultivated land, woodland, mudflat, swamp, and water. The samples must be representative and evenly distributed in the selected area. Different experimental samples are selected by manual visual interpretation method, and the sample separability method is used to check the sample accuracy. Among them, the value of sample separability is between 0 and 2, and the larger the value is, the better the separability is. In this study, kappa coefficient and confusion matrix are used to evaluate the extraction results, and ROI data are used to verify the training accuracy.

The separability tables of training samples and real ROI data are shown in Tables 1 and 2. It can be seen from Tables 1 and 2 that the training and verification samples have good separation, and the separability is higher than 1.9, which can be applied to information extraction and accuracy verification.

Through the real ROI sample data, the confusion matrix, production accuracy, and user accuracy are calculated. The overall kappa coefficient is 0.91, and the classification accuracy is 93%. The confusion matrix of wetland extraction method based on deep learning is shown in Table 3.

The user accuracy and production accuracy calculated by the method proposed in this study are shown in Table 4. The results show that more than 90% of water targets can be identified, and the user accuracy and production accuracy are 99.78% and 91.94%, respectively. The user precision and production precision of swamp, bog, cultivated land and woodland, constructed wetland, construction land, and bare land were 91.04% and 79.65%, 91.04% and 96.61%, 87.06% and 98.64%, 80.96% and 99.23%, 98.60% and 86.76%, 93.23% and 98.73%, respectively. Among them, ponds, constructed wetlands, cultivated land, woodland, and bare land have higher production accuracy. Swamp, bog, construction land, and bare land have higher user accuracy.

### 3.2. Comparison of Accuracy between Different Methods

In this study, decision tree classification, support vector machine (SVM), object-oriented, minimum distance, maximum likelihood, and the methods proposed in this paper are used to carry out comparative experiments in the experimental area. Among them, decision tree classification is mainly to construct the rules of landscape and establish decision tree to extract landscape features. The object-oriented method mainly uses many experiments to determine the best spatial segmentation scale to extract landscape features. SVM, minimum distance, and maximum likelihood methods need to select local samples and determine the field segmentation area. The method proposed in this study mainly uses multiple experiments to divide the optimal grid and identify landscape features and then preset the threshold to extract wet map spots. The results of landscape information extraction using the above methods are shown in Figure 8.

It can be seen from Figures 8 and 9 that although the minimum distance method can extract water information, it is easy to confuse swamp and construction land, and there are many errors and omissions, which is the worst accuracy of the comparison method in this paper. Compared with the former, the accuracy of maximum likelihood method is improved. Although this method improves the identification ability of construction land, it is easy to identify the swamp as an industrial wetland; SVM method is superior to the first two methods, the extraction accuracy of this method has been greatly improved, the classification accuracy of construction land and constructed wetland has been effectively improved, and most of the water features can be extracted; only a few of them are wrong or missing, but it is still easy to confuse swamp and water body. The accuracy of decision tree classification is similar to that of SVM, which is slightly higher by 2.12%, and kappa coefficient is increased by 0.02, but there is still less misclassification in the classification of constructed wetlands. The accuracy and kappa coefficient of object-oriented method are higher than those of the above four methods and are close to SVM and decision tree on the whole.

The accuracy comparison results between various methods are shown in Figure 9. As can be seen from the results in Figure 9, the kappa coefficient of the proposed method is 0.91, which is 0.26, 0.2, 0.1, 0.08, and 0.04 higher than the minimum distance method, maximum likelihood method, SVM, decision tree classification method, and object-oriented method, respectively. The overall accuracy is 93.33%, which is 23.31%, 18.11%, 9.07%, 6.95%, and 4.26% higher than the minimum distance method, maximum likelihood method, SVM, decision tree classification method, and object-oriented method, respectively. The kappa coefficient and the overall accuracy are the best.

## 4. Discussion

Deep learning is the development trend in the era of big data. Academia and even industry pay great attention to deep learning. Deep learning has developed rapidly in intelligent recognition and understanding of voice and image. This paper introduces deep learning algorithm, combined with remote sensing image spectral characteristics, constructs wetland information extraction model based on deep learning, extracts lake wetland information, obtains time series wetland distribution information, uses landscape ecology method to analyze wetland spatiotemporal evolution characteristics, and provides important data support for wetland protection, restoration, and decision-making.

Lake wetland plays a very important role in the whole ecological environment and human sustainable development. Due to the problems of economic development and human destruction, Poyang Lake wetland has gradually deteriorated, so it is necessary to protect and restore the lake wetland. First of all, we should protect the wetland which has been found to prevent further damage. To establish perfect protection measures for lake wetland, according to the factors of complete ecological functions, biodiversity, wetland area size, and so on, we should establish wetland protection areas of various levels, start from small scale, and gradually expand to the whole wetland area. It is very important to establish a scientific and reasonable evaluation system for lake wetland ecosystem. The lake wetland has been destroyed constantly, so it is difficult to provide services for specific decision-making only by understanding the wetland area and distribution from a macro perspective. However, there are still some deficiencies in the assessment of wetland changes from the perspective of landscape ecology. Therefore, it is necessary to establish a scientific and effective wetland ecological evaluation system to provide guidance for the protection and development of lake wetlands. Secondly, the dynamic monitoring system of wetland was established, and the dynamic monitoring of wetland was carried out by using multisource satellite remote sensing image data. The 3S technology was used to obtain wetland information regularly, and the wetland change trend was analyzed and predicted. At present, UAV has developed rapidly and has the characteristics of fast time and high resolution, which can also be used to make up for the lack of satellite remote sensing image monitoring of wetlands. At the same time, we should establish a sound wetland information management system to scientifically guide and manage the development, protection, and restoration of wetlands.

Wetland protection not only needs the management and promotion of national government, but also needs the participation of every citizen. To strengthen the publicity of wetland environmental protection, we can not only use TV, but also use network we media and other new communication means to strengthen the publicity of wetland protection, so that more people know about wetlands and attach importance to wetlands. The importance of wetlands should be publicized regularly in schools to establish awareness of wetland protection. Public lectures on the importance of wetland environment can also be held in residential areas, community activity centers, street offices, and other places. Increase investment in wetland protection, and actively carry out research on wetland protection. The lack of funds restricts the work of wetland protection and restoration. At present, many wetland protection areas and wetland investigation and monitoring are difficult to carry out because of the lack of funds, the infrastructure has not been established, and many wetland dynamic monitoring research, wetland protection, and restoration projects are difficult to implement. Therefore, increasing capital investment is conducive to the wetland protection and restoration work. At the same time, increasing scientific research efforts of wetland will provide more detailed understanding of wetland functions, benefits, types, and other aspects and provide scientific basis and decision support for wetland protection, management, utilization, and wetland restoration.

There are still some problems in the process of establishing the deep convolutional neural network model, which need to be further studied and improved in the following aspects: (1) the training and learning of wetland recognition model based on deep learning needs a large number of wetland samples, and the more the number of samples, the better the training effect of model learning. However, due to the limited time, the data in this paper is limited to Landsat series images, and the sample database needs to be further expanded. (2) Due to time and data reasons, only the first-level wetland category is extracted, but not the second-level wetland category. It is necessary to further improve the wetland classification and corresponding samples in the future.

## 5. Conclusion

In this study, aiming at the planning of modern urban landscape, a landscape information extraction model based on multiscale CNN is proposed, and the network quantitative effect of the model is analyzed. The results show that the overall kappa coefficient is 0.91 and the classification accuracy is 93% by calculating the confusion matrix, production accuracy, and user accuracy. The proposed method can identify more than 90% of the water targets, and the user accuracy and production accuracy are 99.78% and 91.94%, respectively. Compared with the minimum distance method, maximum likelihood method, SVM, decision tree classification method, and object-oriented method, the proposed method improves by 0.26, 0.2, 0.1, 0.08, and 0.04, respectively. The overall accuracy is 93.33%, which is 23.31%, 18.11%, 9.07%, 6.95%, and 4.26% higher than the minimum distance method, maximum likelihood method, SVM, decision tree classification method, and object-oriented method, respectively. The proposed method is obviously better than other methods, and the kappa coefficient and overall accuracy are the best. Due to the limited ability, there is no classification of landscape, so we will pay more attention to the research in the future.

## Figures and Tables

**Figure 1:** The receiving field of image data is imported into CNN to extract information features.

**Figure 2:** Multiscale CNN learning and training structure process.

**Figure 3:** Process of pixel classification in remote sensing image using single CNN.

**Figure 4:** Multiscale CNN structure.

**Figure 5:** Humidity component map after tassel cap change. (a) Original 7, 3, 2 band combination. (b) NDWI grayscale image. (c) *K*-*T* transform humidity component gray scale image.

**Figure 6:** The structure of multiscale CNN.

**Figure 7:** Characteristic maps of various training samples.

**Figure 8:** Comparison of experimental results of 6 different methods. (a) Minimum distance method. (b) Maximum likelihood method. (c) SVM. (d) Decision tree. (e) Object-oriented method. (f) Method of this paper.

**Figure 9:** Accuracy comparison of six different methods.

**Table 1:** Separability of training samples.

Class	Water body	Swamp	Mudflat	Cultivated land and woodland	Constructed wetland	Naked land	Land used for building
Water body	—	1.9999999	1.9999998	2.0000000	1.9999678	1.9999998	1.9888393
Swamp	1.9999999	—	2.0000000	1.9894158	2.0000000	1.9998210	1.9944564
Mudflat	1.9999998	2.0000000	—	1.9999998	1.9999998	2.0000000	1.9998868
Cultivated land and woodland	2.0000000	1.9894158	1.9999998	—	2.0000000	1.9999985	1.9999882
Constructed wetland	1.9999678	2.0000000	1.9999998	2.0000000	—	1.9999936	1.9783966
Naked land	1.9999998	1.9998210	2.0000000	1.9999985	1.9999936	—	1.9674826
Land used for building	1.9888393	1.9944564	1.9998868	1.9999882	1.9783966	1.9674826	—

**Table 2:** Separability of real ROI samples.

Class	Water body	Swamp	Mudflat	Cultivated land and woodland	Constructed wetland	Naked land	Land used for building
Water body	—	1.9999965	1.9999998	1.9999999	1.9893866	1.9999972	1.9997943
Swamp	1.9999965	—	1.9981858	1.9996818	1.9896291	1.9985362	1.9797896
Mudflat	1.9999998	1.9981858	—	1.9999998	1.9999988	1.9993146	1.9999929
Cultivated land and woodland	1.9999999	1.9996818	1.9999998	—	2.0000000	1.9999407	1.9994635
Constructed wetland	1.9893866	1.9896291	1.9999988	2.0000000	—	1.9985980	1.9985970
Naked land	1.9999972	1.9985362	1.9993146	1.9999407	1.9985980	—	1.9788310
Land used for building	1.9997943	1.9797896	1.9999929	1.9994635	1.9985970	1.9788310	—

**Table 3:** Confusion matrix of wetland extraction method based on deep learning.

Class	Water body	Swamp	Mudflat	Cultivated land and woodland	Constructed wetland	Land used for building	Naked land	Total
Water body	6224	23	1	6	511	5	0	6770
Swamp	0	1554	0	336	37	0	24	1951
Mudflat	0	36	2653	0	57	0	0	2746
Cultivated land and woodland	0	6	0	2327	26	0	0	2359
Constructed wetland	14	2	0	1	2837	5	0	2859
Land used for building	0	77	0	3	36	1193	66	1375
Naked land	0	9	0	0	0	7	1240	1256
Total	6238	1707	2654	2673	3504	1210	1330	19316

**Table 4:** Production precision and user precision of wetland extraction method based on deep learning.

Class	User accuracy (percent)	Producer accuracy (percent)	User accuracy	Producer accuracy
Water body	99.78	91.94	6224/6238	6224/6770
Swamp	91.04	79.65	1554/1707	1554/1951
Mudflat	99.96	96.61	2653/2654	2653/2746
Cultivated land and woodland	87.06	98.64	2327/2673	2327/2359
Constructed wetland	80.96	99.23	2837/3504	2837/2859
Land used for building	98.60	86.76	1193/1210	1193/1375
Naked land	93.23	98.73	1240/1330	1240/1256

## Data Availability

The data used to support the findings of this study are available from the corresponding author upon request.
